The article "Exploring the Asymmetric Impact of Public Debt on Renewable Energy Consumption Behavior" was retracted in 2025. Reasons: unreliable results or conclusions; a conflict of interest; concerns about the peer review; concerns about the citations.

# Exploring the Asymmetric Impact of Public Debt on Renewable Energy Consumption Behavior

**DOI:** 10.3389/fpsyg.2022.922833

**Published:** 2022-07-05

**Authors:** Luo Jianhua

**Affiliations:** School of Public Administration, Southwest University of Finance and Economics, Chengdu, China

**Keywords:** public debt, renewable energy consumption, Asia, consumption behavior, asymmetric, corporate

## Abstract

The mounting pollution burden has raised the need for renewable energy demand throughout the world. The study aims to explore the effect of public debt on renewable energy consumption for selected 23 Asian economies for the time period 1990–2019. Long-run empirical findings of the group-wise symmetric ARDL model reveal that increasing public debt results in declining renewable energy consumption. However, findings of the long-run group-wise asymmetric ARDL model reveal that positive shock in public debt reduces renewable energy consumption, and negative shock in public debt results in increasing renewable energy consumption. The economy-wise empirical findings of the FMOLS model reveal that an increase in public debt results in increased renewable energy consumption in nine economies and decreased renewable energy consumption in six economies. The asymmetric FMOLS findings reveal that positive shock in public debt increases renewable energy consumption in nine economies and also decreases renewable energy consumption in nine economies. However, a negative shock in public debt increases renewable energy consumption in 12 economies and decreases renewable energy consumption in 5 economies. Additionally, this research provides numerous policy implications for renewable energy sources in Asian economies. Asian governments should use public debt for the consumption of renewable energy resources.

## Introduction

Environmental degradation has become the major issue of the present world owing to its adverse consequences for human life and biological system and its preservation has become the global policy agenda. The United Nations (UN) has declared “clean energy” as the 17th sustainable development goal (SDG) to cope global environmental problems. Greenhouse gas (GHG) emissions need to be reduced by 45% till 2030 in comparison to 2010 levels, attaining net-zero status about 2050 to maintain the 1.5°C goal (IPCC, 2018). Managing environmental issues require substituting non-renewable energy with renewable energy sources. This substitution, however, faces certain challenges such as start-up costs, infrastructures development, and operational costs. These financial constraints play a conducive role in affecting the energy market (Khan et al., 2021a). Besides, there are some market distortions such as asymmetric information and agency cost which make it expensive to use external finance as compared to internal finance, therefore creating certain financial constraints (Modigliani and Miller, 1959; Lei et al., 2021; Hussain et al., 2022). In such a milieu, it becomes difficult to manage the energy-related project.

The article "Exploring the Asymmetric Impact of Public Debt on Renewable Energy Consumption Behavior" was retracted in 2025. Reasons: unreliable results or conclusions; a conflict of interest; concerns about the peer review; concerns about the citations.

Particularly, the issue of financial constraints is more important for the renewable energy sector as compared to the non-renewable energy sector because the expansion of the renewable energy sector is underdeveloped and going through an early stage of development. Therefore, the deployment of renewable energy sources largely depends upon external financial sources (Hussain et al., 2021; Khan et al., 2022). On the one hand, external financing resolves the financial limitations while on the other hand high cost associated with external financing can have negative effects on the renewable energy sector (Khan et al., 2019; Hashemizadeh et al., 2021; Majeed et al., 2021). These financial challenges require the involvement of the government in the deployment of renewable energy projects. In this regard, the role of public debt becomes conducive to promoting renewable energy deployment.

The literature recommends both negative and positive impacts of public debt on renewable energy consumption (Hashemizadeh et al., 2021). On the one hand, public debt helps the country to finance projects related to renewable energy deployment and development. On the other hand, it can also serve as a barrier to the development of renewable initiatives owing to increasing payment liabilities. In a recent study, Hashemizadeh et al. (2021) unpacked the importance of public debt for renewable energy consumption using a sample of 20 emerging economies over the period 1990–2016. Their results revealed a positive association between public debt and renewable energy consumption. Their findings support the view that public debt is also used for supporting renewable energy projects. Similarly, Florea et al. (2021) attempted to identify the impacts of public finance on renewable energy consumption for 11 emerging economies of the European Union (EU) over the period 1995–2015. They employ fully modified ordinary least squares and use two measures of public finances namely budget deficit and public debt. The empirical outcomes suggest the positive influences of both measures of public finances.

Contrary to this, Katircioglu and Celebi (2018) suggest that financing income growth and energy usage through external debt results in a higher environmental loss. That is, economies (particularly, energy-reliant economies) tend to increase their demand for energy owing to high-income growth influenced by high debt amounts. Similarly, some other researchers also consolidate this viewpoint. Hence, if the external debt is used for investment in heavy industrialization, construction sector, infrastructure development, and real estate projects, the energy demand surges which can have adverse environmental consequences (Sun and Liu, 2020; Bese et al., 2021). In a recent study, Wang et al. (2021) demonstrated that an increase in public debt as a ratio of GDP does not increase consumer preferences for the incorporation of renewable energy in their lives. Akram et al. (2021) linked external debt and renewable energy with environmental quality for 33 severely indebted poor nations. Their results suggest that external debt increases the environmental burden by escalating CO_2_ emissions. Furthermore, they also explored the causal associations between selected variables. Their results confirm bidirectional casualty between extern debt and CO_2_ emission, but no causality is found between external debt and renewable energy consumption.

The article "Exploring the Asymmetric Impact of Public Debt on Renewable Energy Consumption Behavior" was retracted in 2025. Reasons: unreliable results or conclusions; a conflict of interest; concerns about the peer review; concerns about the citations.

Existing studies have considered the concerns regarding renewable energy demand, but these studies have not considered the nexus between public debt and renewable energy demand (Lei et al., 2021; Murshed, 2021; Majeed et al., 2022). Moreover, the current literature have explored the linear association between selected variables and completely ignored the non-linear association between these variables. Additionally, we are unable to found any study estimating the nexus between public debt and renewable energy demand in case of Asian economies. The novelty of present study is that it empirically investigates the impact of public debt on renewable energy demand, especially for Asian economies. The aforementioned discussion suggests that only a few studies have explored the public debt and renewable energy nexus. The studies assume linear associations, ignoring the non-linear hidden effects. The literature suggests both negative and positive influences of external debt on renewable energy consumption. Some studies also declared an insignificant association between these two indicators. In such a situation, further research is required to provide a better understanding of public debt and the renewable energy nexus.

This study contributes to the current literature in different manners. First, this study explores the dynamic associations of public debt with renewable energy consumption using both linear and non-linear ARDL/PMG models for Asian economies covering the period from 1990 to 2019. Second, this study provides empirical evidence for individual countries of Asia in a comparative setting. Third, the empirical literature on public debt and renewable energy consumption nexus lacks consensus that justifies further research. Fourth, this study employs non-linear ARDL to explore both the short- and long-run effects of public debt on renewable energy consumption. The results of this empirical study are helpful for academicians, fiscal managers, development practitioners, and environmentalists.

The article "Exploring the Asymmetric Impact of Public Debt on Renewable Energy Consumption Behavior" was retracted in 2025. Reasons: unreliable results or conclusions; a conflict of interest; concerns about the peer review; concerns about the citations.

This research study focuses on Asian economies owing to their unique socioeconomic profile. Asian economies are among the largest borrowers throughout the world; hence the issue of mounting public debt has become a major concern among policymakers and researchers around the globe. The “global financial crisis 2008” and the “Asian financial crisis 1998” are the major causes behind the significant increase of public debt in these economies. We view Asian economies as a suitable sample based on their significant share in global emissions. The Asian economies emitted 16.75 billion metric tons of CO_2_ emissions into the atmosphere in 2020 (World Bank, 2020). This amount is greater than that of total emissions from all other regions of the world. That is Asia-pacific region is the largest contributor to global emissions in the present world. China and India are ranked among the top polluting economies of the world (Chen et al., 2021; Khan et al., 2021b). The share of alone China in Asia-Pacific and global emissions is 60 and 31%, respectively. Asian economies have a substantial influence on global energy demand and consumption and world ecological balance. Therefore, it is imperative to analyze clean energy determinants for Asian economies.

The study tries to answer these questions: (1) Does public debt lead to an upsurge in renewable energy consumption in the Asian region? (2) Do asymmetries in public debt affect renewable energy consumption behavior in the Asian region? To the authors’ knowledge, no prior study has conducted the association between public debt and renewable energy consumption for Asian economies. Particularly, asymmetric associations are not explored so far. We apply an asymmetric model because in the real-world situation public debt is not symmetric. Few studies focused on public debt and renewable energy nexus, but they did not consider asymmetric associations. When analyzing a fluctuating component like public debt, the use of a non-linear model is more appropriate as compared to the linear models. This study attempts to explore renewable energy consumption determinants with a particular focus on public debt as the driver of renewable energy consumption for Asian economies over the period 1990–2019. Economic progress, environmental pressures, and financial globalization are also incorporated as key determinants of renewable energy consumption. The empirical outcomes of this research will suggest appropriate policy formulation to conserve the environmental quality and sustainable economic performance in selected Asian economies and other developing economies with similar profiles. The results of this empirical research are more valuable for those economies which are prioritizing sustainable usage of public debt.

The article "Exploring the Asymmetric Impact of Public Debt on Renewable Energy Consumption Behavior" was retracted in 2025. Reasons: unreliable results or conclusions; a conflict of interest; concerns about the peer review; concerns about the citations.

## Model and Methods

A moderate level of public debt is significant for economic development. An optimum level of public debt helps promote capital inflow and investment, which positively impact economic activities (Grobéty, 2018). On the other, a higher than optimum level of public debt may reduce private investment and social expenditure (Lora and Olivera, 2007; Mohamed, 2013) while increasing inflation, sovereign risk, and burden on the economy (Cochrane, 2011; Qayyum et al., 2014). Few other empirics have also tried to investigate the impact of public debt on a few other indicators, such as poverty, health, education, innovation, and human rights (Mukherjee, 1987; Wamboye and Tochkov, 2015; Vargas et al., 2016; Khan et al., 2020). Public debt directly impacts human development and can also influence the relationship between renewable energy and human development. Public debt can be used to finance renewable energy projects and energy-efficient and clean green technologies. Conversely, a higher level of public debt may become a hurdle in renewable energy projects and environmentally friendly technologies because a higher level of public debt may induce the government to divert financial resources toward financing the budget deficit. In this study, we aim to analyze whether the effect of public debt on renewable energy consumption in selected Asian economies is symmetric or asymmetric. Our study is attached to Krugman’s theory of debt overhanging. The debt overhanging theory of Krugman (1988) reveals that if the future public debts progressively escalate beyond the repayment ability of the country, then it reduces consumption. To explore the impact of public debt on renewable energy consumption by controlling CO_2_ emissions, GDP per capita, and financial globalization, our study follows Hashemizadeh et al. (2021) and built the following model.


(1) $${\text{REC}}_{\text{it}}=\varphi_{0}+\varphi_{1}\,{\text{Debt}}_{\text{it}}+\varphi_{2}\,{\text{CO}}_{2,\mathrm{it}}+\varphi_{3}\,{\text{GDP}}_{\text{it}}+\varphi_{4}\,{\text{FG}}_{\text{it}}+\varepsilon_{\text{it}}$$

Where renewable energy consumption (REC) is dependent on the public debt (Debt), CO_2_ emissions (CO_2_), gross domestic product (GDP), financial globalization (FG), and randomly distributed error term (ε_*it*_). Coefficient estimates from equation (1) is offered long-run estimates. In order to measure the short-run impacts of public debt, we follow Pesaran et al. (2001) and re-write equation (1) in error-correction formats as follows:


(2) $$\Delta \,{\text{REC}}_{\text{it}}=\alpha_{0}+\sum_{i=1}^{\text{p}}\pi_{\text{i}}\,\Delta \,{\text{REC}}_{\mathrm{it}-i}+\sum_{i=0}^{\text{p}}\psi_{\text{i}}\,\Delta \,{\text{Debt}}_{\mathrm{it}-i}$$

$$+\sum_{i=0}^{\text{p}}\mu_{\text{i}}\,\Delta \,{\text{CO}}_{2,\mathrm{it}-i}+\sum_{i=0}^{\text{p}}\theta_{\text{i}}\,{\text{GDP}}_{\mathrm{it}-i}$$

+∑i=0pλ⁢FGit-ii+ω1⁢RECit-1+ω2⁢Debtit-1

$$+\omega_{3}\,{\text{CO}}_{2,\mathrm{it}-1}+\omega_{4}\,{\text{GDP}}_{\mathrm{it}-1}+\omega_{5}\,{\text{FG}}_{\mathrm{it}-1}$$

$$+\lambda .{\text{ECM}}_{\mathrm{it}-1}+\varepsilon_{\text{it}}$$

Specification (2) is recognized as the panel ARDL method that is proposed by Pesaran and Shin (1995) and Pesaran et al. (1999, 2001). In Equation (2), α_0_ represents the intercept term, εit represents the error term, ω_1_, ω_2_, ω_3_, ω_4_, ω_5_are short-run effects, but π_*i*_, Ψ_*i*_, μ_*i*_, θ_*i*_, and λ_*i*_ are long-run effects in the renewable energy consumption model. The long-run linkage among the variables is confirmed *via* cointegration tests, such as F-statistics and ECM or *t*-test. Our objective in this study is to analyze whether the effects of public debt on renewable energy consumption is symmetric or asymmetric. Most of the macroeconomic series move asymmetrically due to exposure to external shocks, and public debt is no exception; hence, applying the asymmetric analysis is justified. Therefore, our study used the panel NARDL method to examine the short and long-run non-linear relationship among the variables. The study incorporated the Fully Modified OLS (FMOLS) method to examine the country-specific results for the Asian region. Therefore, we also have performed the asymmetric analysis. For asymmetric analysis, we need to break the variable of public debt into its positive and negative components by using the partial sum procedure as given below:


(3) Debt+it=∑n=1t△⁢Debt+it=∑n=1tmax⁢(△⁢Debt+it, 0)

(4) Debt-it=∑n=1t△⁢Debt-it=∑n=1tmin⁢(△⁢Debt-it, 0)

In equations 3 and 4, Debt^+^ only represents the positive changes and Debt^–^ represents the negative changes in the series of public debt. In the next step, we will substitute these partial sum variables in place of original variables, as shown below in equation (5).


(5) $$△\,{\text{REC}}_{\text{it}}$$

=α0+∑i=0pπi⁢△⁢REC-it-i+∑i=0pδ⁢△i⁢Debt+it-i

+∑i=0pϕ⁢△i⁢Debt-it-i+∑i=0pμ⁢△i⁢CO2,it-i+∑i=0pθ⁢GDPit-ii

+∑i=0pλ⁢FGit-ii+ω1⁢RECit-1+ω2⁢Debt+it-1

+ω3⁢Debt-it-1+ω4⁢CO2,it-1+ω5⁢GDPit-1

$$+\omega_{6}\,{\text{FG}}_{\mathrm{it}-1}+\lambda .{\text{ECM}}_{\mathrm{it}-1}+\varepsilon_{\text{it}}$$

Equation (5) can now be called panel NARDL-PMG, an extended version of panel ARDL-PMG. The linear cointegration and diagnostic tests are equally applicable in the non-linear method; therefore, no special treatment is required in the non-linear model. For robustness, the study also applies more advanced and sophisticated panel data techniques like FMOLS. This estimator is highly efficient even in the presence of endogeneity among regressors and serial correlation in error terms (Dogan and Seker, 2016; Khan et al., 2021b). Before applying the FMOLS, the study also incorporated cross-sectional dependence and unit root tests. This study also used the cointegration test.

The article "Exploring the Asymmetric Impact of Public Debt on Renewable Energy Consumption Behavior" was retracted in 2025. Reasons: unreliable results or conclusions; a conflict of interest; concerns about the peer review; concerns about the citations.

## Data

The key aim of the study is to explore the impact of public debt on renewable energy consumption for selected Asian economies for a time period ranging from 1990 to 2019. The Asian regions are facing problems in the consumption of renewable energy sources. Our study has chosen time period from 1990 to 2019 based on the data availability. We selected 23 economies based on the data availability. The list of those economies includes Azerbaijan, Armenia, Bangladesh, China, Cambodia, Georgia, Indonesia, India, Iran, Jordan, Japan, Korea, Rep., Kazakhstan, Malaysia, Nepal, Philippines, Pakistan, Russia, Singapore, Sri Lanka, Turkey, Thailand, and Vietnam. Table 1 displays detailed information regarding symbols, definitions, and sources of data. Renewable energy consumption is measured as total consumption of energy from nuclear, renewables, and other sources in quad btu, and this data is extracted from Energy Information Administration (EIA). Data on government debt is sourced from the IMF and it is measured as central government debt in percent of GDP.

**TABLE 1:** Data and sources.

Variables	Symbol	Definitions	Sources
Renewable energy consumption	REC	Total energy consumption from nuclear, renewables, and other (quad Btu)	EIA
Government debt	Debt	Central government debt, total (% of GDP)	IMF
CO_2_ emissions	CO_2_	CO_2_ emissions (kt)	WDI
GDP per capita	GDP	GDP per capita (constant 2010 US$)	WDI
Financial globalization	FG	Financial globalization index	Swiss economic institute

The rising significance of plummeting CO_2_ emissions to combat worldwide environmental change encourages economies to endorse environmental protection and to adopt more renewable energy sources (Saidi and Hammami, 2015; Chen et al., 2021). Bamati and Raoofi (2020) claim that GDP per capita exerts a different impact on renewable energy consumption depending on their level of development. Literature highlights that financial globalization is an imperative determinant of renewable energy consumption (Murshed et al., 2021). A high level of financial globalization can transfer funds to the renewable energy industrial sector in an effective manner. Although GDP and financial globalization and CO_2_ emissions are closely linked with renewable energy consumption, their impact has not been yet discovered in the existing literature. Hence, the present study incorporated the role of all three variables as control variables in the analysis. Data series for CO_2_ emissions and GDP per capita (constant 2010 US$) have been taken from WDI. However, data for the financial globalization index is gathered from the Swiss economic institute.

The article "Exploring the Asymmetric Impact of Public Debt on Renewable Energy Consumption Behavior" was retracted in 2025. Reasons: unreliable results or conclusions; a conflict of interest; concerns about the peer review; concerns about the citations.

## Empirical Results and Discussion

Table 2 reports the results of the cross-sectional dependence test for the selected variables. The test outcome suggests that public debt, REC, CO_2_, GDP, and FG are cross-sectionally dependent. Therefore, second-generation panel unit root tests are conducted which accommodate cross-sectional dependency. In this regard, the CADF and CIPS panel unit root tests are employed to evaluate the extent to which the variables are non-stationary. The results are reported in Table 3. The CADF test outcome suggests that REC, public debt, and GDP are integrated at first difference while CO_2_ and FG are level stationery. Similarly, the CIPS test outcome shows that REC, public debt, and GDP are stationary at their first differences while CO_2_ and FG are level stationery. Thus, both tests declare similar outcomes suggesting that our selected variables have a mixed order of integration. In this case, a suitable estimation approach is ARDL-PMG.

**TABLE 2:** Cross-sectional dependence tests.

	Friedman’s test			Pesaran’s test			
	Cross sectional independence	Off-diagonal elements	Prob.	Cross sectional independence	Off-diagonal elements	Prob.
REC	168.2***	0.599	0.000	18.32***	0.599	0.000
Debt	75.87***	0.471	0.000	6.744***	0.471	0.000
CO2	97.29***	0.569	0.000	13.05***	0.569	0.000
GDP	121.8***	0.393	0.000	13.35***	0.393	0.000
FG	116.3***	0.379	0.000	15.59***	0.379	0.000

***p < 0.01.

**TABLE 3:** Panel unit root tests.

	CADF			CIPS		
	I (0)	I (1)	Decision	I (0)	I (1)	Decision
REC	0.741	−22.11***	I (1)	–0.123	–5.613***	I (1)
Debt	–0.443	−18.90***	I (1)	–1.614	–5.048***	I (1)
CO2	−2.109**		I (0)	−1.881*		I (0)
GDP	0.823	−12.21***	I (1)	–0.042	–3.667***	I (1)
FG	−3.673***		I (0)	−2.142***		I (0)

***p < 0.01.

Table 4 reports the results of ARDL-PMG and NARDL-PMG for renewable energy consumption (REC) and public debt (debt) nexus. Panel A of Table 4 reports long-run results. The results show that public debt exerts a positive and significant influence on REC. Particularly, a one percent increase in public debt will decrease REC by 0.109%. This finding supports the idea that public debt supports such projects which rely on non-renewable energy sources. This finding is consistent with Wang et al. (2021). Furthermore, this result is consistent with the study of Akram et al. (2021) which has demonstrated that external debt increases the environmental burden by escalating CO_2_ emissions in 33 heavily indebted poor countries over the period 1990–2015. This finding is inconsistent with Florea et al. (2021) who showed the favorable effects of public finance on renewable energy consumption for 11 emerging economies of the European Union (EU) over the period 1995–2015. Since their study focuses on EU economies while our study has focused on Asian economies such inconsistency suggests that Asian economies are not sustainably using their public debt.

The article "Exploring the Asymmetric Impact of Public Debt on Renewable Energy Consumption Behavior" was retracted in 2025. Reasons: unreliable results or conclusions; a conflict of interest; concerns about the peer review; concerns about the citations.

**TABLE 4:** Results of ARDL-PMG and NARDL-PMG.

	ARDL-PMG				NARDL-PMG			
	Coefficient	S.E	t-Stat	Prob.*	Coefficient	S.E	t-Stat	Prob.*
**Long-run**								
DEBT	−0.109***	0.024	4.454	0.000				
DEBT_POS					−0.526***	0.054	9.736	0.000
DEBT_NEG					−0.403***	0.044	9.222	0.000
CO_2_	0.279***	0.040	6.937	0.000	0.602***	0.106	5.671	0.000
GDP	0.115***	0.027	4.259	0.000	0.221*	0.125	1.661	0.101
FG	0.040	0.026	1.518	0.130	0.094	0.080	1.187	0.236
**Short-run**								
D (DEBT)	−0.204**	0.096	2.120	0.034				
D [DEBT(–1)]	−0.143**	0.072	1.979	0.049				
D [DEBT(–2)]	0.100	0.069	1.442	0.150				
D(DEBT_POS)					−0.508***	0.100	5.100	0.000
D(DEBT_NEG)					–0.154	0.170	0.906	0.366
D(CO_2_)	0.683	0.483	1.412	0.159	0.282**	0.129	2.180	0.029
D[CO_2_(–1)]	−0.346	0.514	0.674	0.501				
D(GDP)	0.710	0.613	1.157	0.248	0.909*	0.499	1.822	0.069
D[GDP(–1)]	0.111	0.261	0.424	0.672				
D(FG)	−0.120	0.111	1.087	0.278	–0.077	0.085	0.902	0.367
D[FG(–1)]	−0.147	0.167	0.882	0.379				
C	–0.088	0.140	0.630	0.529	–0.250	0.189	1.323	0.187
**Diagnostics**								
Log likelihood	1909.9***				1791.8			
ECM(–1)	−0.423***	0.065	6.480	0.000	−0.507***	0.099	5.100	0.000
Hausman-test	1.035				1.356			
Kao-cointegration	−3.687***				−3.998***			

***p < 0.01; **p < 0.05; and *p < 0.1.

The effect of CO_2_ emissions on REC is positive and significant. The coefficient of CO_2_ implies that a one percent incline in CO_2_ emissions will enhance REC by 0.279 percent. This finding implies that increasing carbon emissions in the atmosphere put pressure on the use of renewable energy sources. Our findings infer that environmental pressure stimulates renewable energy consumption. This outcome gets support from the study of Wang et al. (2020), who documents that environmental apprehensions are prominent for the increase in renewable energy consumption. The effect of GDP emissions on REC is also positively significant. The coefficient of GDP suggests that a one percent incline in GDP emissions will enhance REC by 0.115 percent. This finding suggests that with increasing GDP, the residents of an economy value more environmental amenities and show their willingness to pay for the environment. In this situation, the demand for REC tends to increase. This finding is consistent with Florea et al. (2021) who demonstrated that GDP has a positive and significant influence on REC in 11 emerging economies of the EU from 1995 to 2015. However, this finding is not consistent with Hashemizadeh et al. (2021), who demonstrated a bidirectional association between GDP and REC. The likely reason could be the difference between selected countries for analysis. Our finding is consistent with Alvarado et al. (2020) and Ehigiamusoe and Dogan (2022), who denoted that high-income economies have a high trend of renewable energy consumption in comparison with low-income economies. Ergun et al. (2019) also support our finding by arguing that GDP can prompt the population to reduce the use of traditional energy sources and stimulate them to adopt more effective options for energy consumption, thus, the proportion of renewable energy consumption rises. Another possible justification is that economies make effort for attaining growth in order to improve their citizen’s quality of life, thus, prompting them to use renewable energy sources to drive green growth (Wei et al., 2022). Finally, the impact of financial globalization (FG), however, turns out to be insignificant. This finding suggests that FG perhaps is not the main drive of REC in Asian economies.

The article "Exploring the Asymmetric Impact of Public Debt on Renewable Energy Consumption Behavior" was retracted in 2025. Reasons: unreliable results or conclusions; a conflict of interest; concerns about the peer review; concerns about the citations.

Panel B of Table 4 reports the short-run results. In the short run, the effect of public debt on REC is negative and statistically significant. Particularly, a one percent increase in public debt will decrease REC by 0.204%. The magnitude of this effect is double in the short run; however, the direction and significance level of the effect remains the same in the short run. Thus, the public debt is negatively associated with REC both in the short- and- long run. Panel C of Table 4 reports the results of diagnostic tests. The ECM value for linear ARDL-PMG entails that the rate of adjustment toward the long-run equilibrium is 42% over each year for sampled Asian countries suggesting that any disequilibrium in the short run will converge in the long run. Kao-cointegration test outcome confirms the presence of co-integration in the model, suggesting that the long-term findings are valid in selected Asian economies. Also, panel C of Table 4 suggests that the log-likelihood ratio test supports the model. However, the Hausman test is not significant.

Our primary focus, in public debt changes and REC analysis, is on asymmetries in the selected Asian economies. Therefore, we examine the asymmetries between public debt changes and REC, both in the short and long run. The last four columns of Table 4 report the results for NARDL-PMG. The results reveal that both positive and negative components of REC exert significant influence on REC. The long-run coefficient of public debt suggests that a one percent increase in public debt will decrease REC by 0.526 percent. This finding is consistent with Akram et al. (2021) and Wang et al. (2021).

The effect of a negative shock in public debt also exerts a negative association with REC. The magnitude of the coefficient for a positive effect is larger than that of a negative shock. The findings on the control variable are similar to the findings for linear ARDL-PMG. That is CO_2_ and GDP exert a positive and significant influence on REC while FG does not exert any significant influence on REC.

The short-run results for positive and negative changes in public debt reveal that their effects are dissimilar. A positive change in public debt leads to a significant change in REC while a negative change in public debt does not exert any significant influence. The long-run coefficient of public debt suggests that a one percent increase in public debt will decrease REC by 0.508 percent. Thus, the magnitude of short and long-run positive changes in public debt remain almost similar. However, for the negative shocks magnitude and significance are considerably changed suggesting an asymmetric association between public debt and REC.

The ECM value for NARDL-PMG entails that the rate of adjustment toward the long-run equilibrium is 51% over each year for sampled Asian countries suggesting that any disequilibrium in the short run will converge in the long run. Kao-cointegration test outcome confirms the presence of co-integration in the model, suggesting that the long-term findings are valid in selected Asian economies. The log-likelihood ratio test and the Hausman test are not significant.

To confirm the robustness of results country-specific analysis is also conducted. Table 5 reports symmetric and asymmetric results of FMOLS long-run. The disaggregated results for a positive shock in public debt reveal that partial sum of positive change in public debt has a negative and significant impact on REC in Azerbaijan, Bangladesh, Cambodia, China, Georgia, India, Jordan, Sri Lanka, and Vietnam while it has a positive and significant impact on REC in Iran, Indonesia, Japan, Korea, Rep., Malaysia, Nepal, Philippines, Russia, and Singapore. However, no significant influence is found for Armenia, Kazakhstan, Pakistan, Thailand, and Turkey. The insignificant impact is consistent with the study of Akram et al. (2021) who did not find any causal relationship between external debt and renewable energy consumption in 33 heavily indebted poor countries from 1990 to 2015.

The article "Exploring the Asymmetric Impact of Public Debt on Renewable Energy Consumption Behavior" was retracted in 2025. Reasons: unreliable results or conclusions; a conflict of interest; concerns about the peer review; concerns about the citations.

**TABLE 5:** Symmetric and asymmetric results of FMOLS long-run (robustness).

	Symmetric estimates with FMOLS				Asymmetric estimates with FMOLS				
	Debt	CO_2_	GDP	FG	Debt_pos	Debt_neg	CO_2_	GDP	FG
Armenia	−0.01	0.01***	0.01***	−0.01***	−0.01	−0.01***	0.02***	0.03***	−0.01***
	(0.63)	(3.04)	(4.86)	(2.73)	(0.17)	(4.35)	(7.27)	(8.18)	(4.81)
Azerbaijan	−0.01	0.01	0.01*	0.00	−0.01***	−0.01***	0.01*	0.01***	0.01***
	(0.02)	(0.46)	(1.71)	(0.15)	(3.22)	(6.05)	(1.79)	(4.09)	(7.12)
Bangladesh	−0.02***	0.02***	0.06***	0.00	−0.03***	−0.01	0.03***	0.07***	0.00
	(5.21)	(8.21)	(12.6)	(0.73)	(4.38)	(1.34)	(4.94)	(10.9)	(0.70)
Cambodia	−0.02*	0.03***	0.00	−0.01**	−0.02***	−0.05***	0.04***	0.01	0.00
	(1.88)	(5.47)	(0.28)	(2.17)	(4.47)	(10.6)	(18.9)	(1.49)	(0.30)
China	−2.82***	7.58***	2.02***	−17.7***	−3.00***	−4.04***	10.5***	12.3***	−13.5***
	(15.6)	(12.4)	(4.04)	(24.1)	(8.69)	(10.8)	(27.8)	(8.15)	(28.9)
Georgia	−0.01*	0.02***	−0.01**	0.05***	−0.01*	−0.01*	0.01***	−0.01**	0.02**
	(1.68)	(6.93)	(2.34)	(5.88)	(1.72)	(1.89)	(5.56)	(3.14)	(2.09)
India	−0.12	0.69	3.19***	−1.04***	−2.29***	−2.56***	0.17	3.28***	−0.28**
	(0.45)	(1.58)	(7.77)	(6.14)	(8.47)	(6.93)	(0.52)	(12.1)	(2.14)
Indonesia	0.09***	0.07***	0.48***	−0.02	0.10***	0.08***	0.12***	0.50***	−0.02
	(13.4)	(5.69)	(23.0)	(1.53)	(13.3)	(9.55)	(4.85)	(3.86)	(1.64)
Iran	0.04***	0.06***	0.13***	0.09***	0.06***	0.01	0.10***	0.19***	0.07***
	(6.08)	(4.29)	(4.48)	(7.17)	(16.6)	(1.04)	(6.16)	(3.15)	(12.5)
Japan	1.61***	9.78***	8.22***	−6.92***	1.61***	9.87*	10.0***	10.2***	−6.99***
	(6.59)	(8.08)	(3.63)	(14.4)	(14.1)	(1.75)	(18.0)	(8.74)	(17.9)
Jordan	−0.01***	0.01***	−0.04***	0.00	−0.01**	−0.02***	0.01**	−0.04***	0.02***
	(6.47)	(6.30)	(7.85)	(0.46)	(2.20)	(16.2)	(5.65)	(14.5)	(6.96)
Kazakhstan	0.01	−0.04**	0.08***	−0.06***	−0.01	0.00	−0.04*	0.08***	−0.06***
	(0.42)	(2.06)	(3.91)	(5.82)	(0.26)	(0.68)	(1.80)	(3.44)	(5.26)
Korea, Rep.	0.40***	−0.08	0.44**	−0.05	0.57***	−1.23***	0.42**	0.40**	−0.41***
	(5.26)	(0.36)	(1.99)	(0.56)	(7.24)	(3.02)	(2.00)	(2.06)	(3.40)
Malaysia	0.06***	0.26***	0.60***	0.10	0.10***	0.03	0.30***	0.58***	0.05
	(4.58)	(10.0)	(15.8)	(1.02)	(2.66)	(1.24)	(8.11)	(15.5)	(0.44)
Nepal	0.00	0.00	0.06***	0.01**	0.02***	−0.01***	0.01***	0.04***	0.01***
	(1.34)	(1.59)	(6.92)	(2.24)	(7.00)	(3.72)	(2.60)	(8.55)	(3.18)
Pakistan	−0.04	0.07***	0.71***	−0.01	−0.04	−0.02	0.06**	0.73***	−0.01
	(1.29)	(2.69)	(10.4)	(0.41)	(1.42)	(0.66)	(2.36)	(11.3)	(0.55)
Philippines	0.01	0.05***	0.08***	0.19***	0.11***	−0.04**	0.03***	−0.07***	0.00
	(0.57)	(3.34)	(2.94)	(3.99)	(3.68)	(2.63)	(11.3)	(10.2)	(0.22)
Russia	0.18***	2.78***	1.95***	−0.21**	0.46***	−0.16***	0.55	−0.13	−0.20***
	(4.66)	(7.36)	(13.2)	(2.46)	(11.3)	(3.52)	(1.29)	(0.51)	(3.79)
Singapore	0.01***	0.00	0.01***	−0.04***	0.01***	0.01***	0.00	0.01***	−0.04***
	(29.2)	(0.53)	(4.46)	(6.94)	(26.7)	(4.68)	(0.24)	(5.21)	(15.9)
Sri Lanka	0.00	−0.03***	0.05***	0.04***	−0.01*	0.02**	−0.03***	0.06***	0.04***
	(0.50)	(16.3)	(7.33)	(10.5)	(1.81)	(2.57)	(16.1)	(11.6)	(7.96)
Thailand	0.02***	0.49***	0.75***	0.18***	0.00	0.28***	−0.17***	0.75***	0.23***
	(2.84)	(22.6)	(7.64)	(5.59)	(0.16)	(9.27)	(3.80)	(29.3)	(5.59)
Turkey	−0.13***	−0.76***	1.67***	−0.13	−0.02	−0.64***	−0.09	1.94***	0.04
	(4.24)	(4.64)	(9.18)	(1.41)	(1.55)	(3.48)	(1.23)	(25.9)	(0.94)
Vietnam	0.03**	1.05	2.43***	−0.14**	−0.56***	−0.11***	−0.99***	1.79***	−0.17***
	(2.33)	(1.51)	(2.10)	(2.32)	(9.55)	(5.78)	(21.9)	(17.1)	(3.68)

***p < 0.01; **p < 0.05; and *p < 0.1.

The article "Exploring the Asymmetric Impact of Public Debt on Renewable Energy Consumption Behavior" was retracted in 2025. Reasons: unreliable results or conclusions; a conflict of interest; concerns about the peer review; concerns about the citations.

The disaggregated results for a negative shock in public debt reveal that partial sum of negative change in public debt has a negative and significant effect on REC in Azerbaijan, Armenia, China, Cambodia, Georgia, India, Jordan, Korea, Rep., Nepal, Philippines, Russia, Turkey, and Vietnam while it has a significant positive effect on REC in Indonesia, Japan, Singapore, Sri Lanka, and Thailand. However, no significant effect is found for Bangladesh, Kazakhstan, Iran, Malaysia, and Pakistan. Thus, a disaggregated analysis also confirms an asymmetric association between public debt and REC.

## Conclusion and Policy Implications

Renewable energy is a vastly debated issue throughout the world as it plays a significant role in the economy’s development and ecological improvement. It is projected that renewable energy will share most of the final energy profile of the world by 2050. Due to the increasing demand for renewable energy in the future, a vast body of literature devoted the validation of various determinants, including foreign trade, environmental pressure, urbanization, and economic growth, etc. However, the research vacuum between renewable energy consumption and public debt nexus is neglected. Although, public debt can be considered as pull and push factors, such as a deterrent to investing in cleaner energy and a source of financing for ecological protection programs. In this perspective, the study aims to explore the impact of public debt on renewable energy consumption for selected Asian economies for time period 1990–2019. The study selected 23 economies on the basis of the availability of data. Long-run empirical findings of the group-wise symmetric ARDL model reveal that increase in public debt results in declining renewable energy consumption. However, findings of long-run group-wise asymmetric ARDL model reveal that positive shock in public debt leads to a reduction in renewable energy consumption and negative shock in public debt results in increasing renewable energy consumption. Economy-wise empirical findings of FMOLS model reveal that an increase in public debt results in increasing renewable energy consumption in 9 economies and decreases renewable energy consumption in 6 economies. The asymmetric FMOLS findings reveal that positive shock in public debt increases renewable energy consumption in 9 economies and also decreases renewable energy consumption in 9 economies. However, negative shock in public debt increases renewable energy consumption in 12 economies and decreases renewable energy consumption in 5 economies.

The article "Exploring the Asymmetric Impact of Public Debt on Renewable Energy Consumption Behavior" was retracted in 2025. Reasons: unreliable results or conclusions; a conflict of interest; concerns about the peer review; concerns about the citations.

Our findings provide some essential policy guidelines. First and foremost, the findings of the study are asymmetric in nature, i.e., both positive and negative changes in public debt move asymmetrically. Therefore, policymakers should treat positive and negative changes differently while considering their effects on renewable energy consumption. Consequently, to promote renewable energy consumption, the policymakers should keep an eye on the public debt, and it should not be allowed to increase by a greater amount. On the other side, a fall or negative change in the public debt could increase renewable energy consumption, but it could lead to a decrease in economic growth because previous findings suggest that a certain amount of public debt promotes economic development. As already discussed, a fall in public debt may slow the pace of economic growth, and the projects of renewable energy sources may also stop due to a lack of financial resources. Asian government should public debt efficiently allocated to environmentally friendly sectors in order to maximize renewable energy consumption. The governments of Asian economies should design suitable energy and economic policies that urge the development of renewable energy consumption for the achievement of environmental and economic sustainability in the Asian region. Moreover, renewable energy consumption is positively affected by an increase in the GDP in selected Asian economies. A rise in GDP provides additional resources in the economy, which allows the government to divert its resources toward the projects such as education, health care, infrastructure, and renewable energy that improve society’s overall wellbeing.

The article "Exploring the Asymmetric Impact of Public Debt on Renewable Energy Consumption Behavior" was retracted in 2025. Reasons: unreliable results or conclusions; a conflict of interest; concerns about the peer review; concerns about the citations.

Due to data constraints, the analysis was limited to only 23 selected Asian economies. Additionally, during the selected time period for analysis, various structural breaks occur in selected economies, but our analysis has not considered these structural breaks. It is suggested for future studies to capture the impact of these structural breaks at the country-level so that more appropriate policies can be designed for each economy. In this study, we aim to investigate the determinants of renewable energy consumption and the role of public debt in this regard. The asymmetric analysis provides more realistic results because most of the macroeconomic variables move in an asymmetric manner. Therefore, future studies should focus more on asymmetric analysis for other countries and regions. Moreover, future studies should also try to analyze the effect of public debt on renewable energy consumption by dividing the countries on the basis of the public debt they owe. Future studies should also consider the asymmetric causality among variables.

## Data Availability Statement

The raw data supporting the conclusions of this article will be made available by the authors, without undue reservation.

## Author Contributions

LJ: confirms sole responsibility for the following: study conception and design, data collection, analysis and interpretation of results, and manuscript preparation.

## Conflict of Interest

The author declares that the research was conducted in the absence of any commercial or financial relationships that could be construed as a potential conflict of interest.

## Publisher’s Note

All claims expressed in this article are solely those of the authors and do not necessarily represent those of their affiliated organizations, or those of the publisher, the editors and the reviewers. Any product that may be evaluated in this article, or claim that may be made by its manufacturer, is not guaranteed or endorsed by the publisher.
